The article "Convolutional Neural Network with Multiscale Fusion and Attention Mechanism for Skin Diseases Assisted Diagnosis" was published in 2022. Journal: Comput Intell Neurosci.

# Convolutional Neural Network with Multiscale Fusion and Attention Mechanism for Skin Diseases Assisted Diagnosis

**DOI:** 10.1155/2022/8390997

**Published:** 2022-06-14

**Authors:** Zhong Li, Hongyi Wang, Qi Han, Jingcheng Liu, Mingyang Hou, Guorong Chen, Yuan Tian, Tengfei Weng

**Affiliations:** ^1^School of Intelligent Technology and Engineering, Chongqing University of Science and Technology, Chongqing 401331, China; ^2^Liquor Making Microbial Application & Detection Technology of Luzhou Key Laboratory, Luzhou Vocational & Technical College, Luzhou, Sichuan 646000, China

## Abstract

Melanoma segmentation based on a convolutional neural network (CNN) has recently attracted extensive attention. However, the features captured by CNN are always local that result in discontinuous feature extraction. To solve this problem, we propose a novel multiscale feature fusion network (MSFA-Net). MSFA-Net can extract feature information at different scales through a multiscale feature fusion structure (MSF) in the network and then calibrate and restore the extracted information to achieve the purpose of melanoma segmentation. Specifically, based on the popular encoder-decoder structure, we designed three functional modules, namely MSF, asymmetric skip connection structure (ASCS), and calibration decoder (Decoder). In addition, a weighted cross-entropy loss and two-stage learning rate optimization strategy are designed to train the network more effectively. Compared qualitatively and quantitatively with the representative neural network methods with encoder-decoder structure, such as U-Net, the proposed method can achieve advanced performance.

## 1. Introduction

Melanoma is one of the most serious skin cancers, causing nearly 60,000 deaths each year [1]. But, fortunately, early detection and effective treatment greatly improve the survival rate of the disease [2]. Dermatoscopy is a mature technology that can visualize the deep image information of the skin. Although effective imaging technology can bring shortcuts to doctors' diagnoses, there are still misjudgments. Dermatologists tend to ignore small targets when diagnosing, which are mostly characterized by weak color features. When the lesion features in the lesion image are obvious, there is often a phenomenon that the edge feature is not obvious. Therefore, manual inspection of the dermoscopy image is error-prone and time-consuming work. In an environment dominated by big data [3–5], it is necessary to develop an automatic system for automatic segmentation and auxiliary analysis of dermoscopy images.

Due to the significant variations and differences in shape, color, and texture of melanoma, automatic melanoma segmentation is still challenging. In addition, some samples may contain artifacts such as hair, ruler markings, and color correction, blurring melanoma lesions and making inspection tasks more difficult. Many algorithms based on deep learning are widely used in image segmentation tasks. They all depend on the characteristics of the sample itself, and the analysis process includes feature extraction and prediction. The most typical deep learning method is the deep neural network based on U-Net [6]. With the help of supervised training, U-Net can learn sample semantics deeply and make a prediction. In recent years, many researchers have focused on U-Net and achieved excellent results. Ghafoorian et al. [7] proposed a multistream network with a multiscale encoder, which can construct multiscale context relations through multiscale feature extraction module. However, due to the shallow network, it is impossible to mine the deep information of the image. Zhou et al. [8] have reconsidered the jump connection, where on the basis of the original context semantic combination, the skip connection was densely connected to narrow the semantic gap between the encoder and the decoder features. Ran Gu et al. [9] proposed a comprehensive attention image segmentation method, which combines the encoder and decoder with the comprehensive attention method to deeply understand the location, channel, and scale information of the lesion area in medical images. Although existing methods have achieved success, they still suffer from the target with a small shape (Figure 1(a)), prominent shape (Figure 1(b)), and edge irregular (Figure 1(c)) in predictions. The relatively low pixel difference between melanoma and nonmelanoma regions confuses CNN models. Targets with small shape have high contrast, which tests the fault tolerance performance of the model in prediction. Targets with prominent shapes have obvious characteristic regions, but on the edge of low contrast, the model is difficult to achieve the shrinkage of edge prediction.

The article "Convolutional Neural Network with Multiscale Fusion and Attention Mechanism for Skin Diseases Assisted Diagnosis" was published in 2022. Journal: Comput Intell Neurosci.

In order to solve the problems of shape difference and edge irregularity mentioned above, we propose an image segmentation model based on multiscale feature extraction (MSF). The model is composed of encoder, decoder, and asymmetric skip connection structure (ASCS). Encoder and decoder are used to analyze the context information of lesion images. ASCS can enhance the connection between encoder and decoder and play the role of information compensation. At the same time, the scSE attention mechanism [10] of fusion space and the channel is embedded, and the multiscale global semantic information extracted by MSF is fused to effectively distinguish the spatial location relationship between lesions and nonlesions.

The model we propose is inspired by U-Net [6], so compared with the baseline network (U-Net), the parameters of our model are greatly reduced. In terms of the segmentation effect of the same target, our model is better than U-Net. At the same time, compared with the existing best-performing method, DeepLap [11], our model also achieves quite good results. According to the above results, our model is suitable for irregular lesion segmentation tasks. Our main contributions to the follow-up work are threefold:

1. We propose a multiscale fusion structure (MSF) is proposed to aggregate the filtering results of different scales by using multilayer channels
2. An effective decoder strategy is proposed, which can combine low-level semantic information with high-level semantic information to ensure the relevance of information
3. An encoder and decoder structure for auxiliary diagnosis of lesion area was proposed, which is effective for the segmentation task of irregular lesion area

The rest of this paper is organized as follows.  Section 2 introduces some related work in this paper.  Section 3 describes our proposed MSFA-Net and its novel components: the multiscale fusion structure in Section 3.1, the asymmetric skip connection structure in Section 3.2, and the decoder in Section 3.3.  Section 4 presents our experimental setup, implementation details, and results compared with the most advanced models. The conclusion of our work is provided in Section 5.

## 2. Related Work

### 2.1. Convolutional Neural Networks for Biomedical Imaging Tasks

With the vigorous development of the big data era [12, 13], deep neural network based on data support has been widely applied to various tasks, such as image segmentation, image classification, and target detection. In recent years, due to the sharp increase in the demand for clinical diagnosis, biomedical image processing methods based on deep learning have emerged endlessly [14]. Full convolutional neural network (FCN) [15] and U-shaped network (U-Net) [6] were the earliest convolutional neural networks used for natural image segmentation and biomedical image segmentation. FCN and U-Net all adopt the segmentation network designed by encoder-decoder structure. The encoder is responsible for feature extraction, and the decoder is responsible for upsampling to obtain a segmentation mask, which is consistent with the size of the input image. The difference between U-Net and FCN is that U-Net also introduces an additional skip connection to stitch the feature map output at each down-sampling stage of the encoder to the corresponding stage of the decoder. Therefore, inspired by the skip connection structure, we combine the asymmetric convolution method to further filter the shallow features in the encoder and transmit them to the decoder for calibration of the recovered features.

The article "Convolutional Neural Network with Multiscale Fusion and Attention Mechanism for Skin Diseases Assisted Diagnosis" was published in 2022. Journal: Comput Intell Neurosci.

In the field of biomedical image analysis, researchers often use prior knowledge of clinical anatomical structure to improve the efficiency of the algorithm. Veni et al. [16] used U-Net combined with the shape prior of the heart to segment the four-chamber structure. Duan et al. [17] proposed the 2.5D feature representation of CMR as the input of FCN and limited the network to refine the segmentation results under a shape constraint. Multiscale feature extraction and aggregation play an important role in improving biomedical image segmentation performance. Ahmad et al. [18] proposed a multiscale hierarchical architecture (MH U-Net), which showed excellent performance in medical image segmentation. MH U-Net was composed of encoder-decoder structure and residual inception. Sinha and Dolz [19] used the guided self-attention mechanism to capture richer context dependencies, so as to overcome the limitations of multiscale information redundancy. Feng et al. [20] proposed a novel context pyramid fusion network (CPFNet) by combining two pyramid modules to fuse global or multiscale context information. CPFNet is composed of multilevel series features with different scales. Different from the existing methods, we propose a biomedical image segmentation (MSFA-Net) method based on multiscale information fusion combined with a convolution neural network and encoder-decoder structure. This method effectively combines different scale information in parallel ways to increase the relevance of local and global information.

### 2.2. Skin Lesion Segmentation

In the previous skin disease segmentation work, Yu et al. [21] proposed a fully convolution residual network (FCRN), which used the characteristics of the residual structure to enhance the identification ability of the network by increasing the depth of the network. Although they could obtain more abundant features, they ignored the global information, making the network lack the overall perception of the lesion image. Therefore, only considering the increase of depth cannot effectively complete the task of lesion image segmentation. Alom et al. [22] proposed the recurrent convolution neural network based on U-Net (RCNN) and the recurrent residual convolution neural network based on U-Net (RRCNN). On the basis of a stacked feature extraction structure, the extracted features are reused to enhance the expression ability of the network to the lesion area. However, RCNN and RRCNN are complex, and their response time is slower than that of U-NET, so they are not suitable for the deployment of medical platforms. Sarker et al. [23] replaced the feature extraction encoder with the pretraining model and then combined four pretraining extended residual networks and pyramid pooling modules. However, integrating multiple methods may lead to a sharp increase in parameters and require more running time to achieve network convergence. Therefore, this is not feasible for medical platforms. In our work, we propose a simple network structure from multiscale, so as to develop a lightweight and fast response model.

The article "Convolutional Neural Network with Multiscale Fusion and Attention Mechanism for Skin Diseases Assisted Diagnosis" was published in 2022. Journal: Comput Intell Neurosci.

### 2.3. CNN with Attention Mechanism

Recently, in computer vision, the attention mechanism played an important role in many scenes. Liang Sun et al. [24] proposed a deep learning framework based on anatomical attention guided for brain ROI segmentation in structural MR images. Ren et al. [25] proposed a new strategy with hard and soft attention modules to solve the segmentation problem of hydrocephalus MR images. Ryo Hasegawa et al. [26] used an attention network to extract feature information from three-phase images for simultaneous detection and segmentation of liver tumors in multiphase CT images. Based on the above research, scSE [10] attention block is introduced to the attention module for different shapes and irregular edge texture problems, in this paper, which has good adaptability, so it is very suitable for our architecture.

## 3. Methods

In this section, we discuss how to extract multiscale features from images using dilated convolution. Then, we explain the role of asymmetric convolution structure in this network. Finally, we also elaborated on the decoder structure.

### 3.1. Multiscale Fusion Structure

In order to obtain better multiscale contextual information of input feature maps, multiple convolutions with different expansion coefficients are used in parallel connections to obtain multiscale features. SPP [27] solved the problem of size change by concatenating mapping features. In addition, channel information cannot be ignored. ASPP used dilated convolution to reflect the importance of channels on the basis of multiscale feature extraction. But the pooling operation of the last layer makes ASPP lose the fine information of the global image, which is very important for skin lesions image segmentation.

In order to solve the above problems, we put forward MSFA-Net shown in Figure 2 to further complete the segmentation task. MSF defines two types of convolution kernels, whose sizes belong to a set *K* = {1,3}; *k*_1_ ∈ *K* and *k*_2_ ∈ *K* are scales of a convolution kernel in longitudinal and transverse, respectively. In Figure 3(a), in order to ensure that the global information of the image is retained, 1 × 1 convolution block is used to traverse pixel by pixel, which is crucial for pixel-level medical image segmentation [28]. Therefore, we set *r*_*i*_={1,3,6,12,18*|i*=1,2,3,4,5}, when *r*_1_=1, we use 1 × 1 convolution block to complete the sampling. In Figure 3(b), we use four 3 × 3 dilated convolution blocks with different dilated rate *r*_*i*_(*i*=2,3,4,5) to obtain the spatial information of image features and increase the number of channels to reflect the spatial position relationship.

The article "Convolutional Neural Network with Multiscale Fusion and Attention Mechanism for Skin Diseases Assisted Diagnosis" was published in 2022. Journal: Comput Intell Neurosci.

Define *X*={*x*_*l*_*|x*_*l*_ ∈ *ℝ*^*H*×*W*×*C*^} as the input of MSFA-Net, where *C*=3, and *Y*={*Y*_*i*_*|Y*_*i*_ ∈ *ℝ*^*D*×*E*×*G*^, *i*=1,2,3,4 or 5} is the output with *G* channels of dilated convolution, where *G*=128, and let *M*=(*M*_*ijg*_)_*k*_1_*k*_2_*G*_ be the 3  *D* convolution kernel. When *k*_1_ × *k*_2_=1 × 1, the process of global feature extraction can be calculated as follows:

(1) $$\begin{array}{c} Y_{1}=\sum_{c=1}^{C}x_{l:,:,c}⋇M_{:,:,g}^{\left(k_{1}\times k_{2}\right)}, \end{array}$$

where ⋇ is the 2  *D* convolution operator, *x*_*l*:,:,*c*_ is a *H* × *W* matrix in *c*-th channel in *x*_*l*_ ∈ *X*, and **M**_:,:,*g*_^(*k*_1_ × *k*_2_)^ is the 3  *D* convolution kernel of *g*-th channel with *k*_1_ and *k*_2_.

The 1 × 1 convolution kernel retains global information and maps the relationship of the three channels of the same pixel into the high-dimensional channel. However, the perception of different pixels in the same channel is very limited [29]. In Figure 3(b), we construct the spatial correlation of neighbor pixels by expanding the scale of the convolution kernel and changing the moving amplitude of extracted features and map this correlation into the channels. Define *α* as the scale, which is a distance of two pixels in transverse or longitudinal in a convolution kernel, and *k*_1_ × *k*_2_=3 × 3. The feature extraction process of dilated convolution can be calculated as follows:

(2) $$\begin{array}{c} Y_{i}=\sum_{c=1}^{C}x_{l:,:,c}⋇M_{:,:,g}^{\left(k_{1}\times k_{2}\right)}\left(\alpha \right), \end{array}$$

(3) $$\begin{array}{c} \alpha =r_{i}-1,i\in \left\{2,3,4,5\right\}. \end{array}$$

After the 3 × 3 dilated convolution, we introduce a 3 × 3 conventional convolution to filter the spatial information. In addition, we have added scSE to each layer to improve fine-grained semantic segmentation. Finally, the results *F*_*i*_ of scSE (I) are calculated as follows:

(4) $$\begin{array}{c} \tilde{Y}=\Lambda \left(F_{1},F_{2},F_{3},F_{4},F_{5}\right), \end{array}$$

where $\tilde{Y}$ is the result of MSF, *i*=1,2,3,4,5, and Λ is the concatenation function based on channel.

The article "Convolutional Neural Network with Multiscale Fusion and Attention Mechanism for Skin Diseases Assisted Diagnosis" was published in 2022. Journal: Comput Intell Neurosci.

### 3.2. Asymmetric Skip Connection Structure

Asymmetric convolutions (AC) are typically used to approximate an existing square-kernel convolutional layer for compression and acceleration [30]. Since the number of AC parameters is small and the effect of feature extraction is analogous to square kernel convolution, AC can effectively replace the original square kernel. Based on the above conclusions, the 1 × 3 convolution kernel can obtain the horizontal spatial relationship in the image according to the direction of the sliding window [31]. Similarly, the direction of 3 × 1 convolution kernel is vertical. The convolution structure with horizontal and vertical parallel design can effectively replace the 3 × 3 square structure in cascades, but the number of parameters is reduced by 33% when the performance is slightly decreased [30]. Inspired by the asymmetric convolution block (ACB) [32], we propose an asymmetric skip connection structure (ASCS) shown in Figure 2, and the structure is a bridge, connecting the input and decoder. The specific information on ASCS is shown in Figure 4.

In the calculation, we adjust the values of *k*_1_ and *k*_2_ in formula (1) and set *G*=3. Then the convolution process can be calculated as follows:

(5) $$\begin{array}{c} Y=\sum_{c=1}^{C}x_{l:,:,c}⋇M_{:,:,g}^{\left(k_{1}\times k_{2}\right)}, \end{array}$$

where *k*_1_ × *k*_2_ ∈ {3 × 3,1 × 3,3 × 1} and *Y* is the result of the convolution operation. In order to reduce overfitting and accelerate the training process, we add batch normalization (*bn*) operation. Subsequently, we use the activation function *ReLU* for linear scaling transformation. The calculation process of *bn* and *ReLU* are as follows:

(6) $$\begin{array}{c} Y^{\prime }=bn\left(Y_{:,:,g}\right)=\left(Y_{:,:,g}-\mu \right)\frac{\gamma }{\sigma }+\beta , \end{array}$$

(7) $$\begin{array}{c} Y^{\prime \prime }=\text{ReLU}\left(Y^{\prime }\right)=\left\{\begin{array}{cc} p, & p>0,\\ 0, & p\leq 0, \end{array}\right. \end{array}$$

where *Y*′ is the result of *bn*; *Y*^″^ is the result of ReLU; *μ* and *γ* are the mean and the standard deviation of channelwise in batch normalization layer, respectively; *σ* and *β* represent the scaling factor and bias, respectively; and *p* is the pixel value in the output matrix *Y*′ of *D* × *E*.

Therefore, we can obtain the corresponding feature mapping *Y*_:,:,*g*_^(3 × 3)^, *Y*_:,:,*g*_^(1 × 3)^, and *Y*_:,:,*g*_^(3 × 1)^ by 3 × 3,1 × 3, and 3 × 1 convolution kernel, respectively, and the calculation of aggregation is as follows:

(8) $$\begin{array}{c} \hat{Y}=Y_{:,:,g}^{\left(1\times 3\right)}\left(Y_{:,:,g}^{\left(3\times 3\right)}\right)*Y_{:,:,g}^{\left(3\times 1\right)}\left(Y_{:,:,g}^{\left(3\times 3\right)}\right), \end{array}$$

where *∗* denotes the Hadamar product and $\hat{Y}$ denotes the result after multiplication. In order to prevent the occurrence of network overfitting, we add the dropout function to lock some weights and limit their updating [33].

The article "Convolutional Neural Network with Multiscale Fusion and Attention Mechanism for Skin Diseases Assisted Diagnosis" was published in 2022. Journal: Comput Intell Neurosci.

### 3.3. Decoder

The decoder in Figure 5 contains two input data. One is the output data $\tilde{Y}$ of the encoder, and the other is the output data $\hat{Y}$ of ASCS.

Firstly, the 1 × 1 convolution kernel is used to linearly combine the high-dimensional channel information for reducing the dimensionality of $\tilde{Y}$. Therefore, the high-dimensional channel can completely map the original plane structure on the single channel [29], and the process can be calculated as follows:

(9) $$\begin{array}{c} {\tilde{Y}}^{\prime }=\text{ReLU}\left(bn\left(\tilde{Y}⋇M_{:,:,g}^{\left(1\times 1\right)}\right)\right). \end{array}$$

Secondly, multiply $\hat{Y}$ with the compressed result pixel by pixel to calibrate the original planar structure as follows:

(10) $$\begin{array}{c} {\tilde{Y}}^{\prime \prime }={\tilde{Y}}^{\prime }\times \tilde{Y}. \end{array}$$

Finally, the three features are concatenated in the channel, namely, the low-level feature $\hat{Y}$, the highly compressed feature ${\tilde{Y}}^{\prime }$, and the calibrated feature ${\tilde{Y}}^{\prime \prime }$. In particular, all three features have the same size so that we concatenate them on the channel to obtain the fusion feature map of *H* × *W* × 3:

(11) $$\begin{array}{c} \dot{Y}=\Lambda \left(\hat{Y},{\tilde{Y}}^{\prime },{\tilde{Y}}^{\prime \prime }\right), \end{array}$$

(12) $$\begin{array}{c} Y_{\text{pred}}=\tilde{\sigma }\left(bn\left(\dot{Y}⋇M_{:,:,g}^{\left(1\times 1\right)}\right)\right), \end{array}$$

where $\dot{Y}$ is the result based on channel concatenate. A 1 × 1 convolution kernel is used for feature filtering again, and a normalization operation is performed. The result of *bn* is input to a sigmoid function $\tilde{\sigma }$ to obtain the pixel-level predict result *Y*_pred_.

### 3.4. Loss Function and Its Optimization

The deep learning neural network model needs limited learning times to fit the training data, so as to achieve the purpose of segmentation. Before training the model, some hyperparameter need to be set, such as learning rate, epoch, batch size, and so on. These parameters play a key role in the network results. Therefore, we propose a learning rate annealing method based on Adam (LRAA), which can adaptively adjust the relationship between learning rate and gradient change according to the change of the loss values of the adjacent two iterations. When our network is trained a certain number of times, the neural network parameters are close to the optimal parameters, that is, the network is more convergent. At this time, the gradient change is weak and needs to be fine-tuned. Therefore, LRAA can adapt to the phenomenon of weak gradient change and achieve high recognition accuracy. In order to represent the LRAA more comprehensively, the training process and optimization process of the neural network are represented by Algorithm 1. In order to accelerate the network fitting, we extracted $\hat{Y}$, ${\tilde{Y}}^{\prime }$, and ${\tilde{Y}}^{\prime \prime }$ as the presegmentation results to compare with the labels *Y*_*label*_ and comprehensively considered their losses. Combined with formulas (8)–(10), their losses can be calculated as follows:

(13) $$\begin{array}{c} f\left(Y_{\text{out}},Y_{\text{label}}\right)=f\left(Y_{\text{pred}},Y_{\text{label}}\right)+\mu f\left(\hat{Y},Y_{\text{label}}\right)+, \end{array}$$

(14) $$\begin{array}{c} \mu +\nu +\xi =1, \end{array}$$

where *f* is the cross-entropy loss function, *Y*_out_ ∈ *ℝ*^*D*×*E*×*G*^ is the output of MSFA-Net, and *Y*_out_ contains $\hat{Y}$, ${\tilde{Y}}^{\prime }$, ${\tilde{Y}}^{\prime \prime }$, and *Y*_pred_. *μ*, *ν*, and *ξ* are loss coefficients, which belong to [0,1].

The article "Convolutional Neural Network with Multiscale Fusion and Attention Mechanism for Skin Diseases Assisted Diagnosis" was published in 2022. Journal: Comput Intell Neurosci.

## 4. Experimental Results

### 4.1. Implementation Details

Our model is developed in Python and implemented in PyTorch. We use a two-class cross-entropy loss function to calculate the loss between the output *Y*_out_ of MSFA-Net and the original labels *Y*_*label*_ and then carry out backpropagation. Training is implemented under the computational specification of 64-bit Windows 10, with Intel i7 processor (3.6 GHz), 32 GB random-access memory (RAM), and NVIDIA Geforce RTX 3090 GPU (24G). Cross-validation is used in the training process to fit the network and data for better prediction results. After the training, we use the validation set to evaluate the optimal model and detect the test set. For the hyperparameter setting, the learning rate *η* is set 10^−4^ in the experiment, the attenuation coefficient *τ* is half of the iteration of training *s*, and *s* = 150.

#### 4.1.1. Images of the Skin Lesion

In this work, we analyze the ISIC2018 [34] melanoma data set and divide the original 2,594 lesions. Given cross-validation, we divide the data set into 1,814 training images, 260 validation, and 520 test.

#### 4.1.2. Data Preprocessing

When original images are loaded, these images will be enhanced by some methods, including random rotation and center clipping in shape to expand the amount of data. At the same time, the label of each image, namely *Y*_label_, also performs the same operation to ensure the accuracy of the segmented target. We carefully compare the differences and connections between the training images, and the color is very different between the skin lesion area and the surrounding normal skin. So we adjusted the color contrast, hue, brightness, and saturation. In addition, since the original size range of images in the ISIC2018 is 720 × 540 to 6708 × 4439 [35], we adjust the size of each image to 224 × 224 and normalize it with mean and standard deviation. The image size for training is 224 × 224 × 3. The output of MSFA-Net is 224 × 224 × 1, which is the same as the *Y*_label_, so it is convenient to compare the pixel difference.

The article "Convolutional Neural Network with Multiscale Fusion and Attention Mechanism for Skin Diseases Assisted Diagnosis" was published in 2022. Journal: Comput Intell Neurosci.

#### 4.1.3. Metric Methods

The pixel-level metric indicators of segmentation accuracy are based on:

(1) Calculate the ratio of intersection and union between predicted segmentation *Y*_pred_ and original label *Y*_label_ as follows:
  (15) $$\begin{array}{c} \text{IoU }=\frac{\left|Y_{\text{pred}}\cap Y_{\text{label}}\right|}{\left|Y_{\text{pred}}\cup Y_{\text{label}}\right|}=\frac{TP}{TP+FP+FN}. \end{array}$$
(2) Set similarity measure between *Y*_pred_ and *Y*_label_ as follows:
  (16) $$\begin{array}{c} \text{ Dice }=\frac{2\left|Y_{\text{pred}}\cap Y_{\text{label}}\right|}{\left|Y_{\text{pred}}\right|+\left|Y_{\text{label}}\right|}=\frac{2\text{TP}}{\text{FP}+2\text{TP}+\text{FN}}, \end{array}$$
where *TP* (*TN*) is the number of pixels correctly predicted and marked as positive (negative). On the contrary, FP (FN) is the number of pixels wrongly predicted and marked as positive (negative). Intersection over union (IoU) and dice similarity coefficient (Dice) are used to evaluate whether each pixel is correctly divided into positive or negative values. Thus, more comprehensive consideration is given to the evaluation results.

### 4.2. Lesion Segmentation from Dermoscopic Images

#### 4.2.1. MSF Based on Different Dilated Rates

We research the feature extraction capability of different dilated rates. As the encoder structure of MSFA-Net, the MSF aims to obtain feature information of different scales, and different scales are determined by different dilated rates. We compare the different dilated rates of multiscale fusion block to obtain a better group of dilated rate as follows:

1. We first select (*r*_1_, *r*_2_, *r*_3_)=(1,2,3) with the maximum covenant of *r*_*i*_ is not greater than 1 [11]. Next, we increase the multiple of *r*_*i*_ based on the size of the convolution kernel, so (*r*_4_, *r*_5_)=(15,21) or (*r*_4_, *r*_5_)=(9,15). As shown in Table 1 and Figure 6, we find that increasing the dilated rate will not bring better results because when the convolution kernel scans the bound of image, the area with padding = 0 will be extracted, which results in inaccurate feature extraction of the convolution kernel.
2. Based on the above experiment, we keep the size of the first layer of the convolution kernel unchanged. And the rates of the remaining four layers are defined as multiples of three, (*r*_1_, *r*_2_, *r*_3_, *r*_4_, *r*_5_)=(1,3,6,12,18). According to Table 1, we find that with the increase in rate *r*_*i*_, the prediction results of lesion area did not become better. When (*r*_1_, *r*_2_, *r*_3_, *r*_4_, *r*_5_)=(1,3,6,12,18), the prediction results of our method for 224 × 224 lesion images are the most friendly.

The article "Convolutional Neural Network with Multiscale Fusion and Attention Mechanism for Skin Diseases Assisted Diagnosis" was published in 2022. Journal: Comput Intell Neurosci.

In the experiment, we add the scSE attention mechanism to different locations in the network to improve the generalization ability of the model. The processing effect in scSE (II) is shown in Figure 6. We obtain three sets of segmentation renderings with different rate combinations. It can be observed that MSF with maximum *r*=18 pays close attention to almost every pixel. MSF not only fully expresses its channel characteristics but also captures more perfect spatial information. Although the larger *r*=21 can also capture the overall contour, in Table 1, the IoU is not as good as *r*=18 as *Y*_label_. it is different from *Y*_label_. Merge ratio is not as good as *r*=18. For the MSF with the maximum *r*=15, the sampling range is not comprehensive enough. In comparison, (*r*_1_, *r*_2_, *r*_3_, *r*_4_, *r*_5_)=(1,3,6,12,18) is more suitable for the segmentation task.

After the above comparison, it can be seen that the introduction of the scSE attention block in our network greatly improves the segmentation accuracy, which is the result of the mutual adaptation of each block.

#### 4.2.2. Compared with SOTA Network

We compare U-NET and the SOTA segmentation network, such as Deeplabv3+ [11]. We train U-Net, Deeplabv3+, and our methods in the same environment, and tested them with the same test sets. There are mainly three types of images: targets with small shape, targets with prominent shape, and targets with edge irregular. We visualized the test results of the three models in Table 2.

At the same time, the comparison results of the experiments are shown in Figure 6(b). It can be observed that:

1. For targets with edge irregular, the performance of U-Net is poor, and our method not only can capture features at various scales but also can retain global initial features based on initial semantic features. It can be seen that MSF can effectively supplement the incomplete feature extraction of cascade convolution structure and is more suitable for irregular edge texture targets.
2. For targets with small and prominent shapes, our network and U-Net can adapt well due to the relatively small change in the marginal area. However, in the segmentation task of large targets, MSFA-Net is very sensitive to sudden changes in the edge and is more adaptable.

The article "Convolutional Neural Network with Multiscale Fusion and Attention Mechanism for Skin Diseases Assisted Diagnosis" was published in 2022. Journal: Comput Intell Neurosci.

#### 4.2.3. Parameters and FLOPs

In the comparison of model parameters, shown in Table 3, we make parallel splicing of dilated convolution structures of different rates and extract features from multiple scales. Compared with the traditional 3 × 3 convolution, the parameters are much less, and in the above decoder structure, we do not do too many upsampling operations but use the initial features to correct the weight relationship between the space and the channel. Our method makes a great contribution to reducing the number of parameters.

## 5. Conclusion and Future Work

We propose a multiscale fusion and attention mechanism image segmentation neural network (MSFA-Net) method, which combines the encoder and decoder structure, and the attention mechanism to provide an auxiliary diagnosis method for medical images with better performance and fewer parameters. Our method can segment lesions of different sizes and irregularities and has good adaptability to sudden changes in texture. Inspired by the existing space and channel attention, we introduce the scSE block, which is more friendly to the segmentation task, to improve our network accuracy. We propose a multiscale fusion block that implicitly fuses feature maps of multiple scales to obtain pixel-level spatial position relationships. The experimental results show that our method has higher accuracy than U-Net, which verifies the effectiveness of the model in this paper. Compared with advanced semantic segmentation models (such as Deepabv3+), MSFA-Net has considerable segmentation accuracy.

To promote the proposed method in the future, we need to increase the data set samples to achieve large data analysis. In addition, the generalization performance of the proposed method for similar data sets needs to be further improved. Therefore, future research should investigate large-scale databases and task-similar data sets and conduct more detailed research on convolution network-based methods.

## Figures and Tables

**Figure 1:** Targets with small shape (a), prominent shape (b), and edge irregular (c). (d), (e), and (f) are their original labels, respectively.

**Figure 2:** MSFA-net.

**Figure 3:** MSF: (a) *r*_1_ and (b) *r*_*i*_ (*i* = 2, 3, 4, 5).

**Figure 4:** A 3 × 3 convolution block for preliminary information filtering, and we connect a 1 × 3 convolution block to a 3 × 1 convolution block in parallel and extract the horizontal and vertical spatial features, respectively.

The article "Convolutional Neural Network with Multiscale Fusion and Attention Mechanism for Skin Diseases Assisted Diagnosis" was published in 2022. Journal: Comput Intell Neurosci.

**Figure 5:** The decoder structure fuses the characteristics of the bridge structure and the encoding structure to form high-level information and finally restores it to the segmentation result.

**Figure 6:** The effects of different interest rate combinations are compared in (a) and our model is compared with other models in (b). (a) Comparison results of different rate combinations (b) comparison results of our method with U-Net and Deeplabv3+.

**Algorithm 1:** LRAA.

**Table 1:** We compare the results of different rate combinations and introduce scSE into the multiscale feature before and after fusion. It is used to compare the impact of single and composite feature maps on global accuracy.

Methods (scSE) (*r*_1_, *r*_2_, *r*_3_, *r*_4_, *r*_5_)	Dice	IoU
MSFA-Net (I and II) (1,2,3,15,21)	0.9066	0.8311
MSFA-Net (I and II) (1,2,3,9,15)	0.9129	0.9112
MSFA-Net (I and II) (1,3,6,12,18)	0.9248	0.8852
MSFA-Net (I) (1,2,3,15,21)	0.9020	0.8374
MSFA-Net (I) (1,2,3,9,15)	0.9026	0.8228
MSFA-Net (I) (1,3,6,12,18)	0.9075	0.8653
MSFA-Net (II) (1,2,3,15,21)	0.8520	0.7972
MSFA-Net (II) (1,2,3,9,15)	0.9199	0.8573
MSFA-Net (II) (1,3,6,12,18)	**0.9271**	**0.9128**

**Table 2:** Comparison of our method with other methods on Dice and IoU.

Method	Dice	IoU
U-Net	0.8777	0.7815
Deeplabv3+	0.9179	0.8752
MSFA-Net (I and II)	0.8248	0.8852
MSFA-Net (I)	0.9075	0.8653
MSFA-Net (II)	**0.9271**	**0.9128**

**Table 3:** Comparison of our method with other methods on DICE and IoU.

Method	Paras (M)	FLOPs (G)
U-Net	9.5	**0.7815**
Deeplabv3+	54.7	0.9
MSFA-Net (I and II)	0.49	3.9
MSFA-Net (I)	**0.16**	3.8
MSFA-Net (II)	0.57	3.9

## Data Availability

The data are available from the corresponding author upon request.
